This article has been retracted.

# BRCA1 inhibits AR–mediated proliferation of breast cancer cells through the activation of SIRT1

**DOI:** 10.1038/srep22034

**Published:** 2016-02-23

**Authors:** Wenwen Zhang, Jiayan Luo, Fang Yang, Yucai Wang, Yongmei Yin, Anders Strom, Jan Åke Gustafsson, Xiaoxiang Guan

**Affiliations:** 1 Department of Medical Oncology, Jinling Hospital, Medical School of Nanjing University, Nanjing 210002, China; 2 Department of Medicine, Rutgers New Jersey Medical School, Newark, NJ 07103, USA; 3 Department of Oncology, The First Affiliated Hospital of Nanjing Medical University, Nanjing 210029, China; 4 Department of Biology and Biochemistry, Center for Nuclear Receptors and Cell Signaling, University of Houston, Houston, TX 77204, USA

## Abstract

Breast cancer susceptibility gene 1 (BRCA1) is a tumor suppressor protein that functions to maintain genomic stability through critical roles in DNA repair, cell-cycle arrest, and transcriptional control. The androgen receptor (AR) is expressed in more than 70% of breast cancers and has been implicated in breast cancer pathogenesis. However, little is known about the role of BRCA1 in AR-mediated cell proliferation in human breast cancer. Here, we report that a high expression of AR in breast cancer patients was associated with shorter overall survival (OS) using a tissue microarray with 149 non-metastatic breast cancer patient samples. We reveal that overexpression of BRCA1 significantly inhibited expression of AR through activation of SIRT1 in breast cancer cells. Meanwhile, SIRT1 induction or treatment with a SIRT1 agonist, resveratrol, inhibits AR–stimulated proliferation. Importantly, this mechanism is manifested in breast cancer patient samples and TCGA database, which showed that low SIRT1 gene expression in tumor tissues compared with normal adjacent tissues predicts poor prognosis in patients with breast cancer. Taken together, our findings suggest that BRCA1 attenuates AR-stimulated proliferation of breast cancer cells via SIRT1 mediated pathway.

The androgen receptor (AR) is a member of the steroid hormone receptor family, which also includes the oestrogen receptor (ER), progesterone receptor (PR), and peroxisome proliferator-activated receptor-γ (PPARγ)^1^. These more recent data demonstrate that AR is expressed in more than 70% of breast cancers and has been implicated in breast cancer pathogenesis^2^,^3^. Multiple epidemiologic studies have demonstrated the increased risk of breast cancer development in postmenopausal women with high estrogen and high androgen levels^4^,^5^. Recently, *in vitro* data have shown that the effects of androgens may be dependent of the expression of AR. Activation of AR with dihydrotestosterone (DHT) in human breast cancer cell lines expressing both ER and AR decreased estrogen-dependent signaling to a similar magnitude as that seen with tamoxifen^6^. Accumulating evidence supports the fact that AR plays a critically important role in the development and progression of breast cancer and may be an independent prognostic factor for breast cancer. A recent meta-analysis of women with early breast cancer showed a better overall survival (OS) and disease-free survival (DFS) irrespective of co-expression of ER^7^. However, it was also reported that AR expression was a significant predictor of worse OS and DFS in both univariate and multivariate analyses of patients with triple-negative breast cancer (TNBC)^8^. TNBC tends to occur in premenopausal women and members of specific ethnic groups and a subset are associated with heritable BRCA1 mutations, whereas BRCA1 dysfunction seems to play a major role in the development and progression of disease^9^,^10^. A study reported a high prevalence of BRCA1 dysfunction in sporadic basal-like breast cancer^11^. We speculated that BRCA1 dysfunction could result in a high expression level of AR in human breast cancer. However, little is known regarding the relationship between BRCA1 and AR expression in the human breast cancer.

Reports have shown that there are a significant number of ER^−^/HER2^+^ breast cancers that express AR and are growth stimulated by androgens^12^. Androgens and AR stimulate oncogenic Wnt and HER2 signaling pathways in ER^−^/HER2^+^ breast cancer, which indicates an intrinsic link between AR and growth factor pathways in ER-negative breast cancer^12^. Moreover, clinical trials of the anti-androgen bicalutamide in ER^−^/AR^+^ metastatic breast cancer are ongoing (NCT00468715). However, it was previously suggested that AR could inhibit endogenous ERα transactivation in ERα-positive breast cancer^6^. The same articles showed that AR is significantly associated with OS in ERα-positive breast cancer but not ERα-negative breast cancer^6^. Elevated AR and reduced ERα mRNA were also reported in tamoxifen-resistant tumors *in vitro* and *in vivo*^13^. AR overexpression rendered ERα-positive breast cancer cells resistant to the growth-inhibitory effects of tamoxifen, whereas treatment with the AR antagonist, bicalutamide, reversed this resistance^13^.

In this study, we evaluated the role of BRCA1 in AR-mediated cell proliferation in human breast cancer tissues and cell lines. We found that AR serves as a downstream mediator of BRCA1 function in tumor suppression through the activation of SIRT1, and that resveratrol inhibited AR–stimulated proliferation by activating SIRT1. Importantly, BRCA1–mediated SIRT1 activation was manifested in clinical breast cancer patients and TCGA database.

## Results

### BRCA1 negatively relates to AR expression *in vitro* and *in vivo*

Recent studies have found that the androgen receptor (AR) is expressed in 60–70% of breast tumors^14^. More recently, attention has focused on the role of AR as a prognostic marker and as therapeutic target in breast cancer^7^,^12^. To investigate the relationship between BRCA1 expression and AR status, immunohistochemical (IHC) staining for BRCA1 and AR was performed on malignant tumor samples from 149 non-metastatic breast cancer patients using a tissue microarray. Representative staining is shown in Fig. 1A,B. Of the 149 tumor tissues, 97 cases (65.1%) and 52 cases (34.9%) expressed BRCA1 at high and low levels, respectively, while 67 cases (45.0%) and 82 cases (55.0%) expressed AR at high and low levels, respectively (Supplementary Table S1). Interestingly, we observed a low level of AR expression in BRCA1-enriched tumors. An inverse correlation between BRCA1 and AR expression was observed in those breast cancer tissues tested (r = −0.216, *P* = 0.008) (Supplementary Table S2). Our published data showed that high BRCA1 expression was associated with better OS^15^. Moreover, we also analyzed the association between AR expression and prognosis of these breast cancer patients, and found that low AR expression was associated with better OS (Fig. 1C, 103.18 vs. 84.71 months; *P* = 0.002). Next, we analyzed published The Cancer Genome Atlas (TCGA) data sets of breast tumors to gain an overall view on AR gene expression across different molecular subtypes in breast cancer. Interestingly, we observed a high level of AR mRNA expression in the 1092 primary tumor tissues, comparing with the 111 normal adjacent tissues (*P* = 0.044, Fig. 1D). Importantly, a significantly elevated AR mRNA expression was found between the 111 paired primary tumor and normal adjacent tissues (*P* < 0.0001, Fig. 1E).

Next, western blots for BRCA1 and AR were performed on extracts of breast cancer cell lines representing different molecular subtypes, namely MCF-7 and T47D (Luminal type, ER^+^/PR^+^/HER2^−^), SK-BR-3 (HER2 enriched, ER^−^/PR^−^/HER2^+^), and MDA-MB-157 (basal type, ER^−^/PR^−^/HER2^−^) transfected with BRCA1 clones. As shown in Fig. 1F, transfection of BRCA1 resulted in a significant decrease of AR protein expression in the cell lines MCF-7, T47D, SK-BR-3 and MDA-MB-157 (Fig. 1G). Taken together, our observation indicated that BRCA1 is negatively related to AR expression *in vitro* and *in vivo*.

### BRCA1 induction inhibits AR expression through the activation of SIRT1

SIRT1 is the mammalian homolog of yeast Sir2 and belongs to the seven-member family of NAD^+^ –dependent type III histone and protein deacetylases^16^. Recent studies have demonstrated that SIRT1 could inhibit AR activity and AR-dependent gene transcription by regulating the acetylation levels of AR gene in prostate cancer cells^17^,^18^. To investigate the role of SIRT1 in BRCA1–mediated AR expression, protein expression analysis of SIRT1, SIRT1 target gene mTOR, and AR target gene Skp2/B in the BRCA1*–*transfected cell lines was performed. As shown in Fig. 2A,B, transfection of BRCA1 resulted in some increase of SIRT1 expression and a significant decrease of mTOR and Skp2/B protein expression in the cell lines MCF-7, T47D, SK-BR-3 and MDA-MB-157, suggesting that BRCA1 could activate the expression of SIRT1 in breast cancer. Analysis of a public database of breast cancer samples identified decreased SIRT1 mRNA levels, increased mTOR and Skp2 mRNA levels in 31 breast cancer cell samples with a BRCA1 mutation, compared with 128 breast cancer cell samples without BRCA1 mutation (Fig. 2C and Supplementary Fig. S1)^19^. Taken together, these data suggest that BRCA1 overexpression inhibits AR expression through activation of SIRT1.

It has been shown that SIRT1 plays a role in many important biological processes, including apoptosis, metabolism, cellular senescence, and aging^20^. Here, we also investigated the effect of SIRT1 on cell proliferation and apoptosis in the cancer cell lines mentioned above. As shown in Fig. 2D,E, cell survivals were significantly decreased, while cell apoptosis were increased. Further investigation as to whether SIRT1 activated mTOR/AR/Skp2 downstream pathway found that ectopic expression of SIRT1 inhibited mTOR, AR and Skp2 expression (Fig. 2F,G). Next, we investigated whether knockdown of BRCA1 could reverse AR expression after SIRT1 over-expression. We detected that the expression of AR was in part reversed after the transfection of siBRCA1 in MCF-7 and MDA-MB-157 cell lines (Fig. 2H,I). Taken together, our results indicate that BRCA1 induction inhibits AR expression through the activation of SIRT1.

### Resveratrol attenuates AR–stimulated proliferation by activating SIRT1

Resveratrol is a well-known agonist of SIRT1^21^. Therefore, we hypothesized that resveratrol could attenuate AR–stimulated proliferation of breast cancer cells. To investigate the effects of resveratrol on cellular proliferation, we analyzed the inhibitory effects of increasing concentrations of resveratrol on MCF-7, T47D, and SK-BR-3 cells by MTT assay. Dose-dependent inhibition of cell proliferation was observed, and cell viability was decreased by about 50% following treatment of cells with resveratrol at 40 μM concentration in breast cancer cell lines MCF-7, T47D and SK-BR-3 (Fig. 3A). Hence, we selected this concentration for further studies of resveratrol. To explore the potential role of resveratrol in the cell proliferation and apoptosis in different time durations, we treated the cells with the selective concentration and samples collected at different time points (24, 36, 48, or 60 h) to determine cell survival rates. As shown in Fig. 3B,C, our data further indicated that resveratrol enhanced apoptosis and inhibited cell proliferation at different time points. To explore the mechanism of resveratrol-induced cell apoptosis, we treated cells with resveratrol for 48 h and harvested total protein to detect relative protein expression. As shown in Fig. 3D,E, resveratrol treatment increased levels of SIRT1, inhibited expression of mTOR, AR and Skp2, further suggesting SIRT1 negatively regulates AR expression. Next, we attempted to investigate whether resveratrol specifically could block AR expression by activating SIRT1. We knocked down SIRT1 in the presence of resveratrol and detected the expression of AR in both MCF-7 and MDA-MB-157 cell lines (Fig. 3F,G). We found that the expression of AR was in part reversed after the transfection of siSIRT1 in MCF-7 and MDA-MB-157 cell lines. Collectively, these data indicated that resveratrol attenuated AR–stimulated proliferation at least in part by activating SIRT1.

### SIRT1 overexpression suppresses tumor growth *in vivo*

Although SIRT1 plays a role in many important biological processes has been demonstrated in various cell lines, there was little direct evidence of the effect of SIRT1 *in vivo*. To further provide *in vivo* evidence for the role of SIRT1 in breast cancer, we used a xenograft mouse model. BALB/c mice were subcutaneously injected with MCF-7 cells and intraperitoneally injected with PBS, 100 μM resveratrol, or 200 μM resveratrol every group. As shown in Fig. 4A,B, resveratrol treatment dramatically decreased tumor growth in a dose-dependent manner, in comparison with the control treatment. Moreover, resveratrol treatment also results in a significantly reduced tumor size and weight (Fig. 4C,D). Thus, SIRT1 overexpression reduces the growth of established breast cancer xenografts. Taken together, these results clearly showed that SIRT1 inhibited breast cancer development through diverse cellular processes.

### BRCA1–mediated SIRT1 activation is manifested in breast cancer patients and TCGA database

A critical question that arises from our *in vitro* data is whether the expression of SIRT1 associates with the prognosis of breast cancer patients, and whether the expression of SIRT1 correlates with BRCA1 in the same specimens as predicted by our hypothesis. To address this question, we used an IHC staining analysis to assess the expression of BRCA1 and SIRT1 in specimens from 149 non-metastatic breast cancer patients using a tissue microarray. Representative staining is shown in Fig. 5A,B. Of the 149 tumor tissues, 68 cases (45.6%) and 81 cases (54.4%) expressed SIRT1 at high and low levels, respectively, respectively (Supplementary Table S1). A significant positive correlation between BRCA1 and SIRT1 expression was identified using the breast cancer tissue-array (r = 0.530, *P* < 0.001) (Supplementary Table S3). In addition, we analyzed the association between SIRT1 expression and prognosis of these breast cancer patients, and found that high SIRT1 expression was associated with better OS (Fig. 5C 101.03 vs. 88.38 months; *P* = 0.025). We also found that higher SIRT1 and lower AR expression have better prognosis than other patients (Fig. 5D 110.00 vs. 72.12 months; *P* < 0.001). Next, we analyzed published TCGA data sets of breast tumors to gain an overall view on SIRT1 gene expression across different molecular subtypes in breast cancer. We also found a significant positive correlation between BRCA1 and SIRT1 expression in this database including 1210 patients (r = 0.077, *P* = 0.007) (Fig. 5E). Interestingly, we also observed a low level of SIRT1 mRNA expression in the 1092 primary tumor tissues, comparing with the 111 normal adjacent tissues (*P* < 0.001, Fig. 5F). Taken together, our observations support the correlation between BRCA1 and SIRT1 expression in breast cancer patients and TCGA database.

## Discussion

In the present study, we evaluated the role of BRCA1 in AR–mediated cell proliferation in human breast cancer tissues and cell lines. We report that a high expression of AR was associated with shorter OS in 149 non-metastatic breast cancer patients. Moreover, we reveal that overexpression of BRCA1 significantly inhibited expression of AR through the activation of SIRT1. Meanwhile, SIRT1 induction or treatment with a SIRT1 agonist, resveratrol inhibited AR–stimulated proliferation in breast cancer cells. Importantly, this mechanism is manifested in the breast cancer patient samples and TCGA database, which showed that low expression of SIRT1 in the tumor tissues compared with normal adjacent tissues and OS was significantly longer in patients with a high expression of SIRT1.

BRCA1 is a tumor suppressor protein with important roles in multiple cellular processes, including DNA damage repair, cell cycle checkpoint control, transcriptional regulation, chromatin remodeling, and apoptosis^22^,^23^,^24^,^25^,^26^. Moreover, BRCA1 plays a critical role in the regulation of homologous recombination (HR)-mediated DNA double-strand break (DSB) repair^27^. BRCA1 interacts with the Mre11/Rad50/Nbs1 complex to regulate end resection activity, and contributes to the activation of HR-mediated DSB repair in the S and G_2_ phases of the cell cycle^28^. In addition, recent studies showed that DHT-bound AR could recruit enzymes capable of inducing DSBs^29^. Haffner *et al.* also reported that androgen signaling promotes co-recruitment of AR and topoisomerase II beta (TOP2B) to the genomic breakpoints sites, triggering recombinogenic AR- and TOP2B-mediated DSBs that are found in DHT-stimulated prostate cancer cells^30^. Findings show that AR activity is induced by DNA damage and promotes expression and activation of a gene expression program governing DNA repair^31^. In the present study, we evaluated BRCA1 inhibited AR–stimulated proliferation of breast cancer cells, suggesting that BRCA1 could also play an important role in the regulation of AR-mediated DSBs in human breast cancer.

SIRT1 is the mammalian homolog of yeast Sir2 and belongs to the seven-member family of NAD^+^ –dependent type III histone and protein deacetylases^16^. It has been shown that SIRT1 plays a role in many important biological processes, including apoptosis, metabolism, cellular senescence, and aging^20^. Recent studies have demonstrated that SIRT1 could inhibit AR activity and AR-dependent gene transcription by regulating the acetylation levels of AR gene in prostate cancer cells^17^,^18^. In addition, SIRT1 antagonists could induce endogenous AR expression and enhance DHT-mediated AR expression^17^,^18^. We further demonstrated that BRCA1 induction inhibits AR expression through the activation of SIRT1 and that overexpression of SIRT1 inhibits AR expression through regulation of the expression of mTOR. These observations were consistent with the report that BRCA1 could bind to the SIRT1 promoter and increase SIRT1 expression in human breast cancer^16^.

Resveratrol, the well-known agonist of SIRT1, attenuates AR–stimulated proliferation at least in part by activating SIRT1. Previous studies have suggested that resveratrol could prevent epigenetic silencing of BRCA1 by the aryl hydrocarbon receptor in human breast cancer cells^32^. Our current study demonstrated that mTOR signaling plays a key role in the regulation of AR expression by BRCA1. However, it was recently reported that the mTOR inhibitor rapamycin impairs recruitment of BRCA1 and Rad51 to DNA repair foci, resulting in significant suppression of HR and non-homologous end joining, two major mechanisms required for repairing DNA DSBs^33^. Therefore, further investigation of the role of mTOR signaling in the regulation of BRCA1-mediated AR–stimulated proliferation is warranted.

Skp2 and its isoform Skp2B have been reported to be overexpressed in a variety of cancer types where they contribute to malignant progression^34^,^35^. High levels of Skp2 protein are associated with ER negativity, low p27 expression, high proliferation rate, and poor survival^36^. Emerging evidence has shown that androgen and the AR are involved in the regulation of Skp2. Recent studies have also shown that the AR is a robust upstream regulator of Skp2 through blocking its D-box-dependent degradation in prostate cancer cells^37^. Here, we showed that overexpression of BRCA1 inhibits expression of Skp2/B, through activation of the SIRT1/mTOR/AR pathway. Coincidentally, some studies have suggested that specific inhibition of the mTOR pathway may significantly down-regulate Skp2 levels in both breast and prostate cancer cells^38^,^39^.

In conclusion, our results to date permit construction of a schematic model demonstrating the critical role of BRCA1 in the regulation of AR–stimulated proliferation of breast cancer cells through the activation of SIRT1 (Fig. 5G). Most importantly, key features of this pathway are manifested in breast cancer patients and TCGA database. Together, our results provide a mechanism that BRCA1 attenuates AR-stimulated proliferation of breast cancer cells via SIRT1 mediated pathway and illustrate the great potential of developing new AR-targeting therapy for BRCA1-mutated breast cancer patients.

## Methods

### Clinical Samples

Breast cancer tissues section containing HBre-Duc150Sur-02 (150 cancer cases) were provided by Outdo Biotech (Shanghai, China). Experiments were approved by the Ethics Committee of Jinling Hospital and were conducted in compliance with the Helsinki Declaration. Histological parameters were determined in accordance with the criteria of the World Health Organization. Pathologic staging was performed in accordance with the current International Union against Cancer tumor-lymph node metastasis classification.

### Immunohistochemistry

One hundred and forty-nine breast tumor tissue samples were deparaffinized in xylene, followed by heat-mediated antigen retrieval using citrate buffer (BioGenex Laboratories, San Ramon, CA, USA). Antibody staining was visualized with DAB (Sigma, D-5637) and hematoxylin counterstain. The percentage of positively stained cells was scored on a scale of 0 to 4 as follows: 0 (<1%), 1 (1–24%), 2 (25–49%), 3 (50–74%), and 4 (75–100%). The staining intensity was scored from 0 to 3 as follows: 0 (negative), 1 (weak), 2 (moderate), and 3 (strong). The scores for percentages of positive cells and staining intensities were then multiplied to generate an immunoreactivity score (IS) for each case. The IS ranged from 0–12 (0, 1, 2, 3, 4, 6, 8, 9, and 12). Cutoff values for this scoring system were assigned as follows: high expression of AR, SIRT1 and BRCA1 were defined as an IS of ≥4 (4, 6, 8, 9, and 12); and low expression was defined as an IS of <4 (0, 1, 2, and 3). Immunohistochemical scoring was performed without prior knowledge of the clinical response. Immunostained sections were scanned using a microscope (Aiovert 200; Carl Zeiss).

### Cell Lines and Animals

Breast cancer cell lines MCF-7, T47D, SK-BR-3, and MDA-MB-157 were purchased in 2014 to 2015 from the Chinese Academy of Science Committee Type Culture Collection Cell Bank (Shanghai, China). Authenticity of these cell lines was done by Chinese Academy of Science Committee Type Culture Collection Cell Bank before purchase by STR DNA typing methodology. No authentication of these cell lines were done by the authors. Cells were cultured in RPMI 1640 or DMEM medium (GIBCO, Gaithersburg, MD, USA) supplemented with 10% FBS and 1% penicillin/streptomycin at 37 °C in a humidified atmosphere containing 5% CO_2_. BALB/c athymic nude mice (female, 4–6 weeks) were purchased from the Department of Comparative Medicine, Jinling Hospital (Nanjing, China), and maintained in a pathogen-free facility. Animal studies were performed in accordance with institutional guidelines.

### Reagents

Resveratrol (Selleck Chemicals, Houston, TX, USA) was dissolved in dimethylsulfoxide (DMSO, Sigma) and stored at −80 °C as a 1 mM stock solution. Cells were plated into 6- or 96-well dishes and treated with designated concentrations of resveratrol for 48 h.

### Plasmids and Transient Transfection

Plasmids pBABEpuro HA Brca1 was a gift from Stephen Elledge (Addgene plasmid # 14999)^40^, and Flag-SIRT1 was a gift from Michael Greenberg (Addgene plasmid # 1791)^41^. The BRCA1 and SIRT1 Small interfering RNA and nonspecific control siRNA were all chemically synthesized by Realgene (Nanjing, China), as listed in Supplementary Table S4. Cells (1 × 10^6^ cells/well) were plated in 6-well plates 24 h prior to transfection. Plasmids were then transfected into cells using TurboFect Transfection Reagent (Thermo Scientific) according to the manufacturer’s protocol. Following incubation at 37 °C for 24 h, cells were collected and lysed to verify the expression of related proteins by western blot analysis.

### Cell Survival Assay

A total of 1 × 10^4^ cells per well were seeded into 96-well plates and incubated with various concentrations of resveratrol or transfected with required plasmids for 48 h. Following addition of 20 μL of 0.5 mg/mL MTT solution (Sigma) to each well, the medium was replaced with 200 μL DMSO after 4 h and vortexed for 10 min. Absorbance was measured at 490 nm with a microplate reader (BIO-RAD, USA) to determine the relative numbers of viable cells. Assays were performed independently three times.

### Apoptosis Analysis

Cells were treated with plasmids for 48 h, then harvested by trypsinization (no EDTA) and washed with phosphate-buffered saline (PBS). Analysis of the cell apoptosis was performed as previously described^42^,^43^. Each sample was tested in triplicate and untreated cells were used as controls.

### Western Blotting

Total protein was extracted using RIPA buffer supplemented with protease and phosphatase inhibitors, with protein concentrations determined using a BCA kit (Thermo Scientific). Approximately 20 μg protein was loaded per lane and separated on a sodium dodecylsulfate-polyacrylamide gel and blotted onto nitrocellulose. Blots were blocked with 5% dry milk in tris-buffered saline/0.1% tween-20 and incubated overnight with a diluted solution of primary antibody at 4 °C, followed by incubation with a horseradish peroxidase-conjugated secondary antibody (1:5000) for 2 h. Antibodies used for western blot were: rabbit anti-BRCA1 antibody (CST9010), rabbit anti-SIRT1 antibody (CST9475), rabbit anti-mTOR antibody (CST2983), rabbit anti-Skp2/B antibody (ab19877, ab68455), and rabbit anti-AR antibody (ab74272). Bands were normalized to GAPDH expression, which was used as an internal loading control. Results from at least two separate experiments were analyzed.

### Xenograft Transplantation

Approximately 5.0 × 10^6^ MCF-7 cells were subcutaneously transplanted into the right side of the posterior flank of nude mice. Tumor growth was examined every other day with a vernier caliper. Tumor volumes were calculated by using the equation: V = A × B^2^/2 (mm^3^), wherein A is the largest diameter and B is the perpendicular diameter. When the average tumor size reached about 100 mm^3^, the tumor-bearing nude mice were given with PBS, 100 μM Resveratrol, and 200 μM Resveratrol through intraperitoneal injection (n = 6 mice per group). After three weeks, mice were euthanized and their tumors harvested.

### Statistical Analysis

SPSS Statistics 19.0 (SPSS Inc.) was used for statistical analysis. Data were analyzed using one-way ANOVA or a Student’s t-test. Data are presented as means ± SD of three independent experiments. The log-rank test was used to assess statistical significance of Kaplan-Meier plots. The chi-square test was used for IHC data. The correlation between BRCA1 and AR or SIRT1 expression level was estimated using Spearman’s correlation analysis. A *P* value of < 0.05 was considered statistically significant. *P < 0.05, or **P < 0.001.

## Additional Information

**How to cite this article**: Zhang, W. *et al.* BRCA1 inhibits AR-mediated proliferation of breast cancer cells through the activation of SIRT1. *Sci. Rep.* **6**, 22034; doi: 10.1038/srep22034 (2016).

## Supplementary Material

Supplementary Information

## Figures and Tables

**Figure 1:** BRCA1 negatively related to AR expression in human breast cancer tissues and cell lines. (**A,B**) Representative immunohistochemical staining of BRCA1 high- and AR low-expression (**A**) or BRCA1 low- and AR high-expression (**B**) in breast cancer patient tissues. (**C**) OS in high and low AR-expressing tumor tissues. (**D**) AR mRNA levels from TCGA database including 111 normal adjacent tissues, 1092 primary tumor tissues, and 7 metastatic tumor tissues. (**E**) AR mRNA expression in the 111 paired normal adjacent and primary tumor tissues. (**F,G**) BRCA1 and AR protein expression levels were determined by western blotting and analyzed by grayscale software following transfection of BRCA1 vector or control vector into MCF-7, T47D, SK-BR-3, and MDA-MB-157 cells, and normalized to GAPDH expression. Data are the mean of three independent experiments. *P < 0.05, as compared with control vector transfected cells.

**Figure 2:** BRCA1 induction inhibits AR expression through the activation of SIRT1. (**A,B**) SIRT1, mTOR and Skp2/B protein levels were determined by western blotting and analyzed by grayscale software following transfection of BRCA1 vector or control vector into MCF-7, T47D, SK-BR-3, and MDA-MB-157 cells, and normalized to GAPDH expression. (**C**) Relative levels of SIRT1, mTOR and Skp2 mRNA in 128 BRCA1 wild type (WT) and 31 BRCA1 mutation (MT) breast cancer tissue samples. Data analyzed using Oncomine (www.oncomine.org) from original published data^19^. (**D,E**) Cell viability was measured by MTT assay, and apoptosis was detected by flow cytometry analysis following transfection of SIRT1 vector or control vector into MCF-7, T47D, SK-BR-3, and MDA-MB-157 cells. (**F,G**) SIRT1, mTOR, AR, and Skp2/B protein levels were determined by western blotting and analyzed by grayscale software following transfection of SIRT1 vector or control vector into the indicated six human cancer cell lines, and normalized to GAPDH expression. (**H**,**I**) SIRT1 and AR protein levels were determined by western blotting and analyzed by grayscale software following treatment with SIRT1 vector and/or transfection with siBRCA1 for 48 h, and normalized to GAPDH expression. Data are the mean of three independent experiments. *P < 0.05, as compared with control vector transfected cells.

**Figure 3:** Resveratrol attenuates AR–stimulated proliferation by activating SIRT1. (**A**) Cell viability was measured by MTT assay following treatment of MCF-7, T47D, and SK-BR-3 cells with resveratrol at indicated concentrations for 48 h. (**B**) Cell viability was measured by MTT assay following treatment with resveratrol at the indicated concentrations, for 24, 36, 48, or 60 h. (**C**) Cell apoptosis was detected by flow cytometry analysis after 40 μM resveratrol treatment. (**D**,**E**) SIRT1, mTOR, AR, and Skp2/B protein levels were determined by western blotting and analyzed by grayscale software following treatment with 40 μM resveratrol for 48 h, and normalized to GAPDH expression. (**F**,**G**) SIRT1 and AR protein levels were determined by western blotting and analyzed by grayscale software following treatment with 40 μM resveratrol and/or transfection with siSIRT1 for 48 h, and normalized to GAPDH expression. Data in are the mean of three independent experiments. Res: resveratrol. *P < 0.05, as compared with untreated cells.

**Figure 4:** SIRT1 inhibits tumor growth in a xenograft mouse model. (**A,B**) Total number of tumors after removal from the mice. (**C**) Tumor growth curve. MCF-7 cells xenograft mouse model was intraperitoneally injected with PBS, 100 μM resveratrol, or 200 μM resveratrol every group. Tumor growth was measured from day two after injecting tumor cells. The error bars represent the standard deviation (SD). (**D**) Tumor weight when the tumors were harvested. The data represent the mean ± SD.

**Figure 5:** High SIRT1 expression is associated with longer OS in breast cancer patients. (**A,B**) Representative immunohistochemical staining of BRCA1 and SIRT high- (**A**) or low-expression (**B**) in the breast cancer patient tissues. (**C**) OS in high and low SIRT1-expressing tumor tissues. (**D**) OS in AR high-/SIRT1 low- or AR low-/SIRT1 high-expressing tumor tissues. (**E**) BRCA1 and SIRT1 expression from TCGA database of 1210 patients’ tissues. (**F**) SIRT1 mRNA levels from TCGA database including 111 normal adjacent tissues, 1092 primary tumor tissues, and 7 metastatic tumor tissues. (**G**) A model showing a BRCA1–SIRT1–AR axis signaling pathway involved in tumor cell survival and proliferation. Our data indicate that resveratrol treatment induces the activity of SIRT1, which inhibits AR and potentially other factors leading to reduced cell proliferation and increased apoptosis.

## References

[b1] OlefskyJ. M. Nuclear receptor minireview series. J Biol Chem 276, 36863–36864 (2001).1145985510.1074/jbc.R100047200

[b2] HallR. E. *et al.* Expression of the androgen receptor and an androgen-responsive protein, apolipoprotein D, in human breast cancer. Br J Cancer 74, 1175–1180 (1996).888340110.1038/bjc.1996.513PMC2075941

[b3] LoiblS. *et al.* Androgen receptor expression in primary breast cancer and its predictive and prognostic value in patients treated with neoadjuvant chemotherapy. Breast Cancer Res Treat 130, 477–487 (2011).2183747910.1007/s10549-011-1715-8

[b4] CauleyJ. A. *et al.* Elevated serum estradiol and testosterone concentrations are associated with a high risk for breast cancer. Study of Osteoporotic Fractures Research Group. Ann Intern Med 130, 270–277 (1999).1006838410.7326/0003-4819-130-4_part_1-199902160-00004

[b5] HankinsonS. E. *et al.* Plasma sex steroid hormone levels and risk of breast cancer in postmenopausal women. J Natl Cancer Inst 90, 1292–1299 (1998).973173610.1093/jnci/90.17.1292

[b6] PetersA. A. *et al.* Androgen receptor inhibits estrogen receptor-alpha activity and is prognostic in breast cancer. Cancer Res 69, 6131–6140 (2009).1963858510.1158/0008-5472.CAN-09-0452

[b7] Vera-BadilloF. E. *et al.* Androgen receptor expression and outcomes in early breast cancer: a systematic review and meta-analysis. J Natl Cancer Inst 106, djt319 (2014).2427321510.1093/jnci/djt319

[b8] ChoiJ. E., KangS. H., LeeS. J. & BaeY. K. Androgen receptor expression predicts decreased survival in early stage triple-negative breast cancer. Ann Surg Oncol 22, 82–89 (2015).2514550310.1245/s10434-014-3984-z

[b9] DiazL. K., CrynsV. L., SymmansW. F. & SneigeN. Triple negative breast carcinoma and the basal phenotype: from expression profiling to clinical practice. Adv Anat Pathol 14, 419–430 (2007).1804913110.1097/PAP.0b013e3181594733

[b10] TurnerN. C. & Reis-FilhoJ. S. Basal-like breast cancer and the BRCA1 phenotype. Oncogene 25, 5846–5853 (2006).1699849910.1038/sj.onc.1209876

[b11] TurnerN. C. *et al.* BRCA1 dysfunction in sporadic basal-like breast cancer. Oncogene 26, 2126–2132 (2007).1701644110.1038/sj.onc.1210014

[b12] NiM. *et al.* Targeting androgen receptor in estrogen receptor-negative breast cancer. Cancer Cell 20, 119–131 (2011).2174160110.1016/j.ccr.2011.05.026PMC3180861

[b13] De AmicisF. *et al.* Androgen receptor overexpression induces tamoxifen resistance in human breast cancer cells. Breast Cancer Res Treat 121, 1–11 (2010).1953333810.1007/s10549-009-0436-8PMC2995248

[b14] NiemeierL. A., DabbsD. J., BeriwalS., StriebelJ. M. & BhargavaR. Androgen receptor in breast cancer: expression in estrogen receptor-positive tumors and in estrogen receptor-negative tumors with apocrine differentiation. Mod Pathol 23, 205–212 (2010).1989842110.1038/modpathol.2009.159

[b15] ZhangW. *et al.* BRCA1 regulates PIG3-mediated apoptosis in a p53-dependent manner. Oncotarget 6, 7608–7618 (2015).2579724410.18632/oncotarget.3263PMC4480703

[b16] WangR. H. *et al.* Interplay among BRCA1, SIRT1, and Survivin during BRCA1-associated tumorigenesis. Mol Cell 32, 11–20 (2008).1885182910.1016/j.molcel.2008.09.011PMC2577018

[b17] FuM. *et al.* Hormonal control of androgen receptor function through SIRT1. Mol Cell Biol 26, 8122–8135 (2006).1692396210.1128/MCB.00289-06PMC1636736

[b18] DaiY. *et al.* Sirtuin 1 is required for antagonist-induced transcriptional repression of androgen-responsive genes by the androgen receptor. Mol Endocrinol 21, 1807–1821 (2007).1750506110.1210/me.2006-0467PMC3839341

[b19] PawitanY. *et al.* Gene expression profiling spares early breast cancer patients from adjuvant therapy: derived and validated in two population-based cohorts. Breast Cancer Res 7, R953–964 (2005).1628004210.1186/bcr1325PMC1410752

[b20] HaigisM. C. & GuarenteL. P. Mammalian sirtuins-emerging roles in physiology, aging, and calorie restriction. Genes Dev 20, 2913–2921 (2006).1707968210.1101/gad.1467506

[b21] HowitzK. T. *et al.* Small molecule activators of sirtuins extend Saccharomyces cerevisiae lifespan. Nature 425, 191–196 (2003).1293961710.1038/nature01960

[b22] MullanP. B., QuinnJ. E. & HarkinD. P. The role of BRCA1 in transcriptional regulation and cell cycle control. Oncogene 25, 5854–5863 (2006).1699850010.1038/sj.onc.1209872

[b23] ZhuQ. *et al.* BRCA1 tumour suppression occurs via heterochromatin-mediated silencing. Nature 477, 179–184 (2011).2190100710.1038/nature10371PMC3240576

[b24] ChapmanM. S. & VermaI. M. Transcriptional activation by BRCA1. Nature 382, 678–679 (1996).875143610.1038/382678a0

[b25] HuenM. S., SyS. M. & ChenJ. BRCA1 and its toolbox for the maintenance of genome integrity. Nat Rev Mol Cell Biol 11, 138–148 (2010).2002942010.1038/nrm2831PMC3899800

[b26] PathaniaS. *et al.* BRCA1 is required for postreplication repair after UV-induced DNA damage. Mol Cell 44, 235–251 (2011).2196323910.1016/j.molcel.2011.09.002PMC3200447

[b27] ZhangJ. & PowellS. N. The role of the BRCA1 tumor suppressor in DNA double-strand break repair. Mol Cancer Res 3, 531–539 (2005).1625418710.1158/1541-7786.MCR-05-0192

[b28] ChenL., NieveraC. J., LeeA. Y. & WuX. Cell cycle-dependent complex formation of BRCA1.CtIP.MRN is important for DNA double-strand break repair. J Biol Chem 283, 7713–7720 (2008).1817167010.1074/jbc.M710245200

[b29] WuD., ZhangC., ShenY., NephewK. P. & WangQ. Androgen receptor-driven chromatin looping in prostate cancer. Trends Endocrinol Metab 22, 474–480 (2011).2188935510.1016/j.tem.2011.07.006PMC3229688

[b30] HaffnerM. C. *et al.* Androgen-induced TOP2B-mediated double-strand breaks and prostate cancer gene rearrangements. Nat Genet 42, 668–675 (2010).2060195610.1038/ng.613PMC3157086

[b31] GoodwinJ. F. *et al.* A hormone-DNA repair circuit governs the response to genotoxic insult. Cancer Discov 3, 1254–1271 (2013).2402719710.1158/2159-8290.CD-13-0108PMC3823813

[b32] PapoutsisA. J., LamoreS. D., WondrakG. T., SelminO. I. & RomagnoloD. F. Resveratrol prevents epigenetic silencing of BRCA-1 by the aromatic hydrocarbon receptor in human breast cancer cells. J Nutr 140, 1607–1614 (2010).2063132410.3945/jn.110.123422PMC3139234

[b33] ChenH. *et al.* The mTOR inhibitor rapamycin suppresses DNA double-strand break repair. Radiat Res 175, 214–224 (2011).2126871510.1667/rr2323.1PMC4412148

[b34] RadkeS., PirkmaierA. & GermainD. Differential expression of the F-box proteins Skp2 and Skp2B in breast cancer. Oncogene 24, 3448–3458 (2005).1578214210.1038/sj.onc.1208328

[b35] GstaigerM. *et al.* Skp2 is oncogenic and overexpressed in human cancers. Proc Natl Acad Sci USA 98, 5043–5048 (2001).1130949110.1073/pnas.081474898PMC33160

[b36] SignorettiS. *et al.* Oncogenic role of the ubiquitin ligase subunit Skp2 in human breast cancer. J Clin Invest 110, 633–641 (2002).1220886410.1172/JCI15795PMC151109

[b37] WangH., SunD., JiP., MohlerJ. & ZhuL. An AR-Skp2 pathway for proliferation of androgen-dependent prostate-cancer cells. J Cell Sci 121, 2578–2587 (2008).1862830410.1242/jcs.030742PMC2729111

[b38] ShapiraM., KakiashviliE., RosenbergT. & HershkoD. D. The mTOR inhibitor rapamycin down-regulates the expression of the ubiquitin ligase subunit Skp2 in breast cancer cells. Breast Cancer Res 8, R46 (2006).1685951310.1186/bcr1533PMC1779462

[b39] LiB. *et al.* Skp2 regulates androgen receptor through ubiquitin-mediated degradation independent of Akt/mTOR pathways in prostate cancer. Prostate 74, 421–432 (2014).2434747210.1002/pros.22763PMC4062570

[b40] CortezD., WangY., QinJ. & ElledgeS. J. Requirement of ATM-dependent phosphorylation of brca1 in the DNA damage response to double-strand breaks. Science 286, 1162–1166 (1999).1055005510.1126/science.286.5442.1162

[b41] BrunetA. *et al.* Stress-dependent regulation of FOXO transcription factors by the SIRT1 deacetylase. Science 303, 2011–2015 (2004).1497626410.1126/science.1094637

[b42] LaiJ. *et al.* Transcriptional regulation of the p73 gene by Nrf-2 and promoter CpG methylation in human breast cancer. Oncotarget 5, 6909–6922 (2014).2507101010.18632/oncotarget.2230PMC4196172

[b43] NieW. *et al.* TXNIP interaction with the Her-1/2 pathway contributes to overall survival in breast cancer. Oncotarget 6, 3003–3012 (2015).2560502110.18632/oncotarget.3096PMC4413633

